RETRACTED

# Design and Implementation of Online Intelligent Mental Health Testing Platform

**DOI:** 10.1155/2022/9270502

**Published:** 2022-02-17

**Authors:** Shengtao Ren, Xiangling Hou, Juzhe Xi

**Affiliations:** Shanghai Key Laboratory of Mental Health and Psychological Crisis Intervention, Affiliated Mental Health Center (ECNU), School of Psychology and Cognitive Science, East China Normal University, Shanghai 200062, China

## Abstract

In order to solve the problems of high misevaluation rate and low work efficiency in the process of mental health intelligent evaluation, a method of mental health intelligent evaluation system oriented to the decision tree algorithm is proposed. First, the current research status of mental health intelligent evaluation was analyzed and the framework of mental health intelligent evaluation system was constructed. Then, the mental health intelligent evaluation data were collected and the decision tree algorithm was used to analyze and classify the mental health intelligent evaluation data to obtain the mental health intelligent evaluation results. Finally, specific simulation experiments are used to analyze the feasibility and superiority of the mental health intelligent evaluation system. The experimental results show that the recall rate of each system increases with the increasing number of iterations, and the system has the highest recall rate. Also, it is stable after the number of iterations reaches 20, with good recall and adaptive scheduling performance. The recall rate of comparison system 1 and comparison system 2 fluctuates greatly, and the recall rate is lower than that of the system in this paper. It is proved that the method of the mental health intelligent evaluation system of the decision tree algorithm can effectively solve the problem and improve the accuracy of the mental health intelligent evaluation. The efficiency of mental health intelligent evaluation is improved, and the system stability is better, which can meet the actual requirements of current mental health intelligent evaluation.

## 1. Introduction

College students are in the late stages of youth development, and their own physical and psychological activities have changed greatly. They often experience more negative emotions, and their self-regulation and self-control abilities are not strong yet; therefore, when dealing with problems such as learning, social interaction, friendship, and love, it often causes intense conflicts of psychological contradictions, resulting in disorders and imbalances in psychological development [1]. As the backbone of the future development of the country and society, college students will have serious consequences if their development is affected by psychological factors. Especially when they leave the campus and enter the society, they are very susceptible to the influence or temptation of various bad factors, which will be a fatal blow to the social groups that cultivate them or their parents and teachers even irrelevant [2, 3].

RETRACTED

In short, the social environment facing college students is constantly changing, and their own learning initiatives, hobbies, academic performances, the expansion of the gap between the rich and the poor in the family, and the pressure of employment competition all have different characteristics in the past. The factors that induce their mental health problems show more complex and diverse characteristics, so it is necessary to use information technology to conduct in-depth research on their mental health problems and explore the intervention model [4, 5]. The combination of psychological problem analysis and data mining technology is to find hidden regularities in a small amount of data on mental health problems. This is a scientific method to improve students mental health diagnosis by using advanced intelligent means [6].

Most of the theoretical methods use traditional classification and association analysis methods to study mental health problems. However, classification and counting need to know the type of data in advance. However, in practice, we cannot know which mental health problems are among the following freshmen, so it is very difficult to obtain the class label in advance [7]. In addition, the number of students with information health problems is a minority compared to the overall total and can be classified as abnormal. The use of anomaly detection technology has a better effect on discovering these individuals. Finding out the related factors that affect the mental health of college students is a significant problem. Through the technique of correlation analysis, discovering the frequent patterns and association rules of psychological problems can understand the causes of college students' mental health problems from a deeper level and eliminate hidden dangers in a targeted manner [8]. Zhang et al. gave a design plan of a data mining system for college students' mental health problems. The main method is to use the ID3 algorithm to build a decision tree for classification mining and the Apriori algorithm for association rule mining. From the perspective of this article, there is a good background in psychology research, but the data it uses are only obtained from the mental health test questionnaire, and the object of the study is only students of a certain grade in the author's school. Moreover, the literature is not in-depth enough to master the technology of data mining and the experimental tests conducted [9]. Alghamdi et al. used the decision tree C4.5 algorithm to establish a mental health assessment model, constructed a decision tree, and predicted mental health by extracting rules. This document only uses a relatively simple classification algorithm for applied research and does not involve the analysis of related factors that form college students' mental health problems [10]. Manna and Misra studied the mental health of vocational students in their master's thesis, the main data mining algorithms used are the ID3 decision tree algorithm and the Apriori association rule algorithm to analyze the inherent relationship between psychological problems and their attributes. In addition, the document also studied the psychological data analysis of multidimensional data warehouse model of higher vocational students and designed a prototype system with VB. From the literature, its work is more systematic and comprehensive, but its biggest shortcoming is that it does not analyze the results of data mining, so there is no regular knowledge [11]. In order to improve the effectiveness of mental health intelligent evaluation, a mental health intelligent evaluation system based on a decision tree algorithm is proposed, which can effectively promote the information management of the system, solve the old problems of traditional system resources, give full play to the advantages of the Internet, create a new Internet environment, and effectively solve the psychological problems of contemporary people.

RETRACTED

## 2. Mental Health Intelligent Evaluation System

### 2.1. The Overall Structure of the Mental Health Intelligent Evaluation System

In order to enable people to have an accurate understanding of their own mental health and at the same time to promote the scientific and informatization of mental health guidance, a mental health intelligent evaluation system based on the decision tree algorithm is constructed, and scientific mental health evaluation tools are used to comprehensively and objectively reflect the user's mental health level. The overall structure of the system is shown in Figure 1 [12].

The mental health intelligent evaluation system based on the decision tree algorithm mainly includes four modules: basic information management module, evaluation test question management module, evaluation result analysis module, and personal psychological evaluation module. The basic information management module provides users with the functions of personal information input and evaluation type selection, and after the user submits the above options, the evaluation test question management module provides users with corresponding evaluation test questions. The test questions are divided into three types: selection, question and answer, and test paper composition. After the user selects the assessment item, the system provides the corresponding test questions for them; after the user completes the answer, the evaluation result and corresponding processing are given; and after the answer is completed, the submitted test result can obtain the corresponding detailed single or multiple analysis in the evaluation result analysis module [13].

RETRACTED

### 2.2. Functional Modules of the Mental Health Intelligent Evaluation System

#### 2.2.1. Data Management Section

The basic information management module is the basic function in the system, and its main function is to manage the basic information in the system. This module has the function of personal information synchronization and evaluation type management. The former can synchronize the personal information filled by the user, accurately track the user's real-time personal situation, and ensure the accuracy of the subsequent evaluation of the system in this article. The latter can uniformly manage all the evaluation types in this system, such as mental health, emotional behavior, interpersonal communication, and add or delete evaluation types according to user needs. In the process of using the system, users have multiple types of choices, high versatility, powerful overall system functions, and can be widely used in the crowd [14].

#### 2.2.2. Evaluation Test Question Management Module

The evaluation test question management module is an important part of the system, and the quality of the evaluation test questions seriously affects the correctness of the evaluation results. This module mainly includes three types of test questions: choice test questions, essay test questions, and test paper grouping questions. The forms of multiple-choice questions are multiple-choice questions, which can be single-choice or multiple-choice questions, and there is a strong correlation between the test questions. Answers are made in the evaluation test questions through selection, and according to the different answers selected by the user, jumped to different question types to complete the answer, and the answer points of each question are different. The question form of the question and answer test is a question and answer question, which is designed according to the different types of assessment. The test question form of the test paper combination combines the choice test and the essay test, and it combines the abovementioned two test question types with different evaluation types, jumps to the multiple-choice or essay based on the user's answer, and stops the jump after jumping to the essay. The system can effectively reduce the user's psychological precautions through the skipping of thinking in the choice of test questions, increase their interest in testing, make the test easier to be accepted by them, and get a deeper understanding of the user's psychological state through quiz questions [15].

RETRACTED

#### 2.2.3. Evaluation Result Analysis Module

The evaluation result analysis module is responsible for statistically analyzing the psychological evaluation results of users, discovering the psychological problems of users and grasping their psychological conditions at the first time, and providing help to users. This module can provide users with the analysis results of a single evaluation, comprehensive analysis results of multiple evaluations, function of filling in analysis opinions, and effectively and timely obtain user feedback information on the evaluation results [16].

#### 2.2.4. Personal Psychological Assessment Module

The personal psychological assessment module is the main module in this system, which highlights the significance of this system for users. The evaluation item selection part provides users with all the evaluation items of the system. Users can select the evaluation items according to their own needs. The evaluation question call function can select the corresponding evaluation questions according to the selected evaluation items for users to evaluate and automatically save the answer results of users and give corresponding scores. Finally, the evaluation results of users are processed through the evaluation result processing function, and the processing results are fed back [17].

### 2.3. Analysis of Personal Mental Health

#### 2.3.1. Data Mining Process

The client software of the system uses the method of psychological evaluation data mining to realize the analysis of evaluation results, process the obtained user evaluation result data, and establish a database, through the decision tree algorithm to analyze its evaluation results and get an evaluation. Psychological assessment data mining includes extracting data from the database, cleaning the data, selecting the mining mode, and outputting the results. The complete data mining process is shown in Figure 2 [18]. In this paper, an initial dataset is established by using the user's answer results. After data integration, data extraction, data cleaning, and data conversion, a mental health assessment dataset to be mined is obtained. The decision tree algorithm is applied in the mining process, and the classification of data is obtained through the mining results. Thus, the specific classification of users' mental health status can be obtained.

RETRACTED

#### 2.3.2. Decision Tree Algorithm

The decision tree algorithm is an inductive learning algorithm, which is a classification rule obtained by inducing a set of chaotic examples based on examples, and the rules are represented by a tree structure. When the decision tree deals with the classification problem, it mainly includes two steps: the first is to generate a decision tree classification model through the learning and training set; the second is to classify unknown types of samples through the model. In the classification process of a certain type of sample, the root node is the starting point and a leaf node is the end point, and the sample attributes are gradually tested in the downward direction of the branch. The system applies the C4.5 decision tree algorithm, and the split index is the information gain rate. It solves the problem of bias in selecting value multiattribute when applying information gain to select test attributes [19]. The definition formula of information gain rate is

(1) $$\begin{array}{c} \text{GainRatio}\left(S,A\right)=\frac{\text{Gain}\left(S,A\right)}{\text{SplitInformation}\left(S,A\right)}, \end{array}$$

where Gain (*S*, *A*) is the information gain of attribute *A* and SplitInformation (*S*, *A*) is the breadth and uniformity of splitting the sample set *S* according to the attribute *A*. The decision tree C4.5 algorithm is used to classify the data of the mental health intelligent assessment to provide data support for the system in this paper.

(2) $$\begin{array}{c} \text{SplitInformation}\left(S,A\right)=-\sum_{i=1}^{n}\frac{\left|S_{i}\right|}{S}\log_{2}\left(\frac{\left|S_{i}\right|}{S}\right). \end{array}$$

In the process of decision tree generation, the most important thing is to determine the split target. In order to determine the split index in the C4.5 algorithm, it is necessary to compare the size of the attribute information gain rate in each training sample data and select the attribute with the largest information gain rate and higher than or equal to the average value of all attributes as a branch node of the decision tree. For the existence of continuous descriptive attributes, the continuity needs to be segmented to obtain a discrete set of intervals [20]. Discretization methods include

(1) The continuity attribute *A* of the value of the discretized continuous interval. The samples of training set *S* are arranged according to the numerical values of continuous attributes in descending order. The minimum and maximum values in the interval are assigned to MIN and MAX, respectively, and the value sequence of attribute values is {*A*_1_, *A*_2_,…, *A*_*n*_}.
(2) Let *A*_*i*_ be the equal division point. If there are *N* equal division points in the interval [MIN, MAX], calculate in order, and the formula for the *i*-th equal division point is
  (3) $$\begin{array}{c} A_{i}=\frac{\text{MIN}+i*\left(\text{MAX}-,\text{MIN}\right)}{N}, \end{array}$$
where *i*=1,2,…, *N*.
(3) Calculate the information gain values in the interval value [MIN, *A*_*i*_][*A*_*i*_, MAX] and compare them with *N* − 1 dividing points.
(4) Let the segmentation threshold of the continuity attribute *A* be the segmentation point with the maximum information gain rate *A*_*k*_, divide the data set on this basis, and set the attribute values in [MIN, *A*_*k*_] and [*A*_*k*_, MAX].

According to the abovementioned discretization method, the information gain rate of all attributes in the candidate attribute set is solved, and the test attribute is the attribute with the largest information gain rate. All possible values in the sample set were used to divide the sample to obtain several subsample sets, and the same method was used to continue to divide all the subsample sets, until they cannot be divided and the decision tree is generated. When using the C4.5 algorithm to generate a decision tree, the selected target class affects the determination of each class. Entropy needs to be used when evaluating the decision tree to get

(4) $$\begin{array}{c} S=-\sum_{i}\left(P_{i}*\log\;P_{i}\right). \end{array}$$

Information gain is the effective reduction of information entropy. According to the information entropy, the variable level used for classification can be determined. If there are two classes of class *A* and class *B* in the training set *S*, and they, respectively, include *x* and *y* records belonging to class *A* and class *B*, then the formula for determining the total amount of information for a certain record in the training set *S* is

(5) $$\begin{array}{c} \text{Info}\left(S\right)=\text{Info}\left(S_{a},S_{b}\right)=-\left(\frac{x}{x+y}.\;\log\frac{x}{x+y}+\frac{y}{x+y}.\;\log\frac{y}{x+y}\right). \end{array}$$

Suppose variable *C* is the root node of the decision tree, and the subclass of the training set *S* is {*S*_1_, *S*_2_,…, *S*_*k*_}, then *S*_*i*_(*i*=1,2,…, *k*) includes *x*_*i*_ and *y*_*i*_ records belonging to class *A* and class *B*, respectively. Get the information volume formula classified in all subcategories:

(6) $$\begin{array}{c} \text{Info}\left(C,S\right)=\sum_{i=1}^{k}\frac{x_{i}+y_{i}}{x+y}\text{Info}\left(S_{iA},S_{iB}\right). \end{array}$$

Suppose variable *C* is the classification node of the decision tree and its information increment value is the largest among all variable information increment values, then, the information increment formula of variable *C* is

(7) $$\begin{array}{c} \text{Gain}\left(C\right)=\text{Info}\left(S\right)-\text{Info}\left(A,S\right). \end{array}$$

Then, the information gain function is defined as

(8) $$\begin{array}{c} \text{Gain}\left(D,S\right)=\text{Info}\left(S\right)-\text{Info}\left(D,S\right),\\ \text{Info}\left(S\right)=I\left(P\right)=I\left(P_{1},P_{2},\ldots P_{k}\right)=I\left(\frac{\left|D_{1}\right|}{\left|S\right|},\frac{\left|D_{2}\right|}{\left|S\right|},\ldots ,\frac{\left|D_{k}\right|}{\left|S\right|}\right)\\ =-\left(P_{1}*\log\;P_{1}+P_{2}*\log\;P_{2}+\cdots +P_{k}*\log\;P_{k}\right),\\ \text{Info}\left(D,S\right)=\overset{n}{\underset{i=1}{\sum }}\frac{\left|S_{i}\right|}{\left|S\right|}\text{Info}\left(S_{i}\right). \end{array}$$

RETRACTED

## 3. Simulation Experiment

### 3.1. Interface of Mental Health Intelligent Evaluation System

The system platform uses the SQLServe database, which has multiple functions, mainly including data confidentiality, integrity, which can ensure the security of the user data. In terms of specific structure, security functions, and channel adaptability, it has the characteristics of standardization, multipolarization, and diversification. The current interface of the system stays in the management interface of the question and answer test, the user can directly enter the options that need to be viewed, and can directly delete the evaluation record. The operation is convenient, and the user has a high degree of freedom.

### 3.2. Validity Test of This System

200 employees of this unit were randomly selected as experimental subjects, the psychological state of college students evaluated by this system and professional psychologists was compared, and the results are shown in Figure 3. According to Figure 3, the psychological evaluation results of the system in this paper are basically consistent with those of professional psychologists, which prove that the system in this paper is not only effective but also has very good evaluation results. At the same time, the number of employees with neurasthenia accounted for the largest proportion, the number of employees with obsessive paranoia and emotional instability were 27% and 22%, respectively, and the number of neurotic and sensitive in communication was less, which was due to the work pressure and competitive pressure of the unit. These employees can effectively reduce the proportion of the number of psychological problems after a period of mood relief according to the results of the system, which proves that the system in this paper is practical and can provide users with effective solutions to psychological problems.

RETRACTED

### 3.3. Data Processing Efficiency Test of Mental Health Evaluation System

In order to verify the data processing efficiency of the system, the mental health service system for the elderly based on Internet technology and the automatic mental health evaluation system for online forum users based on multifeature fusion are used as the comparison systems. Comparison system 1 and comparison system 2 are used to represent the data processing time results as shown in Figure 4. Analyzing Figure 4, we can see that the data processing time of the system has been lower than that of the other two systems. As the amount of data continues to increase, the data processing time of the three systems has changed. The data processing time of the comparison system 1 and the comparison system 2 increases sharply with the increase of the amount of information, and the fluctuation range is large and the stability is poor. The increase in the data processing time of the system is small, the curve is smoother, and the stability is good, after the data volume reaches 5 × 103 GB. The data processing time gradually stabilizes, which proves that the system in this paper has high data processing efficiency and strong stability.

### 3.4. Mental Health Evaluation Accuracy Test

Different noises were added to the three systems to evaluate the mental state of employees, and the accuracy of the mental health evaluation of the three systems was tested, and the results are shown in Table 1. It can be seen from Table 1 that with the continuous increase of noise, the mental health evaluation accuracy of the three systems has decreased, but the mental health evaluation accuracy of the system has been above 90%. In addition, the accuracy rate is not much lower and is relatively stable, while the mental health evaluation accuracy of the other two systems is less than 88%. It shows that the different noise of the three systems has the least influence on the mental health evaluation accuracy of the system in this paper, and the system in this paper has good antinoise performance and high mental health evaluation accuracy.

### 3.5. Mental Health Evaluation Stability Test

The information recall rate can be used to verify the system's data scheduling capability. The higher the recall rate, the more stable it is and the better the system's data scheduling capability. The information recall rate of the three systems was tested in the psychological evaluation, and the results are shown in Figure 5. Figure 5 shows the recall rate of three kinds of system with the increasing number of iterations and ascension, and the recall rate of system 3 proposed in this paper is the highest. After smooth and good recall and adaptive scheduling performance comparison, the number of iterations reaches 20. The recall rate of system 1 and system 2 fluctuates greatly, and the recall rate is lower than that of system 3 proposed in this paper.

RETRACTED

## 4. Discussion

We considered the three languages of Python, NET, and JAVA and finally chose JAVA. Although both Python and Net can develop web projects, JAVA's j2ee architecture is perfect and the web ecology is better, so JAVA was chosen. On the basis of the JAVA language, the back-end uses the MVC mode and uses the MVC development architecture that comes with the Spring framework because Spring is a nonintrusive framework that can minimize the dependence of application code on the framework. The data control layer uses MyBatis, combined with Alibaba's Druid connection pool, which can greatly improve the performance of JAVA applications, while reducing all resource usage and connection creation time. The database uses MySQL of Alibaba Cloud Data. Because MySQL is open source and small in size, the database application and creation can be easily completed in the RDS console. The RD instance can be ready and put into use within a few minutes, and all instances can be managed uniformly. For efficient development, traditional jsp web pages are abandoned, and front-end and back-end development are used. The front-end interface uses HTML and CSS, and JavaScript front-end and back-end separation will increase the front-end work pressure, and reduce the workload of the background. The background does not care about the business realization of the front desk and does not care about the page realization of the front desk. The static interface uses the bootstrap grid layout, and the front-end and back-end interactions use ajax asynchronous requests to obtain the back-end data. The data processing usesjQuery, and the data display layer uses Vue.js because Vue only focuses on the view layer, which can greatly reduce the cost of front-end development, and the front-end and back-end development will not disturb each other.

## 5. Conclusion

In order to improve the effectiveness of mental health intelligent evaluation, a mental health intelligent evaluation system based on the decision tree algorithm is constructed, which can fully help users understand their own mental health, solve their psychological problems, and enhance self-awareness. In order to make the system more functional and have better development, it is also necessary to improve the analysis of system evaluation results and the situation of system data loss during a power failure, increase the system's data backup and recording functions, solve the problem of wasted storage space, and improve the system's functions.

RETRACTED

## Figures and Tables

**Figure 1:** General structure drawing.

**Figure 2:** Psychological assessment data mining flowchart.

**Figure 3:** Comparison results.

**Figure 4:** Data processing time of the three systems.

**Figure 5:** Comparison of recall rates of three systems.

**Table 1:** Mental health assessment accuracy of the three systems.

Noise (dB)	20	40	60	80
System	93.46	92.10	92.74	91.06
Comparison system 1	88.06	87.74	87.73	85.98
Comparison system 2	81.78	81.69	81.02	80.37

## Data Availability

The data used to support the findings of this study are available from the corresponding author upon request.
